# Effect of Different Glucose Monitoring Methods on Bold Glucose Control: A Systematic Review and Meta-Analysis

**DOI:** 10.1155/2022/2851572

**Published:** 2022-06-18

**Authors:** Yeling Wang, Congcong Zou, Han Na, Weixin Zeng, Xiaoyan Li

**Affiliations:** ^1^Department of Radiotherapy, The First Affiliated Hospital of Hainan Medical University, Haikou, Hainan 570102, China; ^2^Reproductive Medicine Center, The First Affiliated Hospital of Hainan Medical University, Haikou, Hainan 570102, China; ^3^Department of Endocrine, The First Affiliated Hospital of Hainan Medical University, Haikou, Hainan 570102, China

## Abstract

**Objective:**

To evaluate the effectiveness of different glucose monitoring methods on blood glucose control and the incidence of adverse events among patients with type 1 diabetes mellitus.

**Methods:**

Using the method of literature review, the databases PubMed, Cochrane, and Embase were retrieved to obtain relevant research literature, and the selected studies were analyzed and evaluated. This study used Cochrane software RevMan5.4 to statistically analyze all the data.

**Results:**

A total of 15 studies were included in this study, including 10 randomized controlled trials and 5 crossover design trials, with a total of 2071 patients. Meta-analysis results showed that continuous blood glucose monitoring (CGM) could significantly reduce the HbA1c level of patients, weighted mean difference (WMD) = −2.69, 95% confidence interval (CI) (-4.25, -1.14), and *P* < 0.001 compared with self-monitoring of blood glucose (SMBG). Meanwhile, the incidence of severe hypoglycemia in the CGM group was significantly decreased, risk ratio (RR) = 0.52, 95% CI 0.35-0.77, and *P* = 0.001. However, there was no statistical difference in the probability of diabetic ketoacidosis between CGM and SMBG groups, RR = 1.34, 95% CI 0.57-3.15, and *P* = 0.5.

**Conclusion:**

Continuous blood glucose monitoring is associated with lower blood glucose levels than the traditional blood glucose self-test method.

## 1. Introduction

Diabetes, as a new global epidemic, has been increasing worldwide in recent years [1]. Diabetes is one of the most common chronic diseases in China, with a high prevalence rate of 12.8% [2]. Meanwhile, it also has a high incidence. Diabetes is divided into type 1 diabetes and type 2 diabetes. Type 1 diabetes is also known as insulin-dependent diabetes mellitus, which occurs primarily in children and adolescents and requires insulin to restore the blood glucose level. Although the incidence rate of type I diabetes is lower than type 2 diabetes, research suggested that type I diabetes has a higher economic cost to the national health care system than type II [3]. The increased financial burden may relate to the reliance on insulin therapy and the occurrence of serious complications [4]. Insulin treatment can effectively decrease blood sugar. Monitoring blood glucose levels is also very important to keep the blood glucose level at a normal level [5, 6].

The detection of blood glucose is helpful to early identify patients with hypoglycemia, evaluate the degree of glucose metabolism disorder, and reasonably formulate personalized blood glucose management plans for patients. However, the traditional self-monitoring of blood glucose (SMBG) method often cannot provide real-time blood glucose data and cannot give early warning of asymptomatic blood glucose abnormalities [7]. Continuous glucose monitoring (CGM) is a dynamic glucose monitoring method that includes an inserting subcutaneous sensor, which can automatically measure the individual interstitial glucose level all day and understand the patient's blood glucose fluctuation by providing an ambulatory glucose profile (AGP) [8]. At present, there are several main types of CGM systems: retrospective CGM (r-CGM), real-time blood glucose monitoring (rt-CGM), and intermittent scanning CGM (isCGM). Each system is slightly different in function [9]. However, the actual effect of CGM on blood glucose control in type 1 diabetes mellitus is uncertain. To further evaluate the effectiveness of CGM and SMBG in maintaining glycemic control among patients with type 1 diabetes, this study will conduct a quantitative meta-analysis by retrieving the latest published clinical studies.

## 2. Method

### 2.1. Bibliography Retrieval

PubMed, Cochrane Library, and Embase were searched from January 2015 to April 2022. Search terms and keywords included “type 1 diabetes OR insulin dependent diabetes OR IDDM OR T1DM OR autoimmune diabetes OR” AND “continuous glucose monitor∗ OR CGM” AND “blood glucose self monitor∗ OR SMBG.”

### 2.2. Literature Screening

Inclusion criteria: (1) the subjects were diagnosed with type 1 diabetes mellitus and were receiving intensive insulin therapy, with a study period of at least 8 weeks. (2) The study must be a two-arm study. The experimental group adopts continuous blood glucose monitoring, and the control group adopts traditional self-blood glucose monitoring; (3) the literature type was a randomized controlled study; (4) the study included at least one of the following outcomes: HbA1c level, severe hypoglycemia (SH), and diabetes mellitus (diabetic) ketoacidosis (DKI). The literature language, publication date, or impact factors were not limited.

Exclusion criteria: (1) news reports, expert opinions, critical literature, and abstracts; (2) republished literature; (3) unable to obtain enough literature to analyze the data.

### 2.3. Document Data Extraction

The literatures were screened and the data extraction was done by Wang and Li independently. The content includes: publication date, author's name, study type, patient inclusion criteria, number of patients, subject characteristics, data results and other information. If there were questions or differences in the literature screening and extraction process, a third researcher assisted in resolving and deciding through discussion at the meeting if necessary.

### 2.4. Literature Quality Evaluation

The quality of the included literature was evaluated according to the risk bias evaluation tool in the Cochrane manual. The evaluation contents include (1) whether the random allocation method is appropriate, (2) whether the random allocation scheme is hidden, (3) researchers and subjects were blinded, (4) blind evaluation of research results, (5) whether the result data is complete, (6) whether there are selective reports of results, and (7) whether there are other sources of bias. The evaluation results were divided into high, low, and uncertain risks. Two researchers independently evaluated the quality of the included literatures and then crosschecked. If there was any difference, both parties discussed it to reach an agreement or ruled by the third researcher.

### 2.5. Statistical Method

This study used Cochrane software RevMan5.4 to statistically analyze all the data. The counting data were statistically described by calculating risk ratio (RR) value and 95% confidence interval (CI), and the measurement data were statistically described by weighted mean difference (WMD) and 95% CI. It was considered statistically significant when *P* < 0.05 using a fixed-effect model or random-effect model. The Chi-square test was used to test the heterogeneity between different studies. When the *I*^2^ corrected by degrees of freedom was more than 50%, it was considered heterogeneous, and the random effect model was used. When *I*^2^ corrected by degrees of freedom is ≤50%, it was considered that there was no heterogeneity, and the fixed effect model was adopted. The potential publication bias was estimated by funnel plot.

## 3. Results

### 3.1. Literature Search Results

In this study, 2124 relevant literatures were obtained through database retrieval. After the retirement, collected literatures were deduplicated by EndNote X9 management software. They were screened through reading topics and abstracts according to the predetermined inclusion and exclusion criteria and then further read the full text for rescreening. Finally, 15 literatures meeting the criteria were included. The specific screening process and results are shown in Figure 1.

### 3.2. Basic Characteristics and Quality Evaluation of Literature

According to the inclusion and exclusion criteria, a total of 15 studies were included. The basic information of the included literature is shown in Table 1. The published time was from 2015 to 2022. The included literature is relatively new. The literature types were prospective clinical trials, including 10 randomized controlled trials and 5 cross-design trials. The study population included people from the United States, the United Kingdom, Switzerland, the Netherlands, and China. The 15 studies included 2071 patients with type 1 diabetes. Most of the continuous blood glucose monitoring methods in the intervention group were real-time blood glucose monitoring, including 11 using RT-GCM, 2 using intermittent scanning CGM, 1 using personal continuous blood glucose monitoring, and 1 using rapid blood glucose monitoring. The insulin regimen included MDI, CSII, and MDI/CSII. The age of patients included adolescents, middle-aged, and elderly, but almost all were under the age of 50. The longest duration of diabetes was about 37 years. The course of each study was mainly 24/26 weeks. Cochrane risk bias assessment tool was used to evaluate the included literature. Only one literature was high-risk, three were uncertain, and the rest were low risk. It was considered that the quality of the included literature was high.

### 3.3. Meta-Analysis Results

All 15 studies reported the HbA1c level of patients after the intervention of CGM and SMBG. The heterogeneity test result *I*^2^ was 73%, which had great heterogeneity. Therefore, the random effect model was used to merge the data. The results of the meta-analysis are shown in Figure 2. Compared with SMBG, CGM could significantly reduce the HbA1c level of patients. The combined result is WMD = −2.69, 95% CI (-4.25, -1.14), and *P* < 0.001. The publication bias of the included studies was detected. The results showed that the included literatures were symmetrically distributed around the combined effect of WMD value. The HbA1c level funnel is shown in Figure 3. It was considered that there was no publication bias.

12 studies reported severe hypoglycemic events among patients after the intervention of CGM and SMBG. The heterogeneity test result *I*^2^ was 23%, and there was no heterogeneity. Therefore, the fixed-effect model was used to merge the data. The results of the meta-analysis are shown in Figure 4. Compared with SMBG group, the incidence of severe hypoglycemic events in CGM group was significantly lower, RR = 0.52, 95% CI 0.35-0.77, *P* = 0.001. The included studies were tested for publication bias. The results are shown in Figure 5. It was considered that there was no publication bias.

The 11 studies reported the risk of diabetic ketoacidosis after CGM and SMBG intervention. The heterogeneity test result *I*^2^ was 0%, and there was no heterogeneity. Therefore, a fixed-effect model was used to merge data. Meta-analysis showed no statistical difference in the probability of occurrence of diabetes ketoacidosis between the CGM group and the SMBG group, RR = 1.34, 95% CI 0.57-3.15, and *P* = 0.5, respectively. The meta-analysis results showed no significant difference in the probability of occurrence of diabetic ketoacidosis. The results are shown in Figure 6. The included studies were tested for publication bias. The results are shown in Figure 7. It was considered that there was no publication bias.

## 4. Discussion

Diabetes, as one of the most common chronic diseases in the country, brings severe illness and financial burden to patients and families. Type 1 diabetes mellitus is dependent on insulin therapy, but this treatment may cause severe hypoglycemia. Therefore, it is essential to maintain the blood glucose level at an average level through real-time monitoring. HbA1c is the gold standard for assessing glycemic control and an alternative indicator [25] for evaluating the risk of long-term diabetes complications. CGM can play an early warning role among patients' blood glucose values as a dynamic blood glucose monitoring method. However, there is still some controversy about the actual effect of CGM on variables such as HbA1c. This study was conducted to analyze and discuss the three indicators of HbA1c level reduction, the incidence of severe hypoglycemia, and diabetes ketoacidosis before and after the intervention.

The results showed that the CGM group decreased by 2.69 mmol/mol at the HbA1c level compared with the SMBG group. Although the reduction was up to 5 mmol/mol, the decrease in HbA1c level is enough to reduce the risk of diabetes complications to a certain extent [13]. In addition, patients with high HbA1c levels often have macrovascular risks. Reducing HbA1c levels can effectively reduce the incidence of cardiovascular disease and death [26]. Compared with the SMBG group, the risk of severe hypoglycemic events in the CGM group was reduced by 48%, which is inconsistent with the results of other meta-analyses [6, 27]. This difference may be related to inconsistent criteria for determining adverse events. Still, the latest published clinical trial [15] showed that CGM could effectively reduce the occurrence of severe hypoglycemic events. There is no difference between the two methods in the incidence of diabetic ketoacidosis. This study indicated that the probability of occurrence of diabetic ketoacidosis was about 1.3%. The incidence of diabetic ketoacidosis was rare. The results of this study are for reference only. Further studies on the effects of CGM on diabetic ketoacidosis are needed.

Some previous studies are consistent with our research direction. Maiorino et al. [28] noted that CGM could benefit patients with diabetes. In particular, this study highlights the advantages of CGM in controlling HbA1c control over time frames. Langendam et al. [29] pointed out that the evidence for the effectiveness of CGM is limited. Previous studies overstated his effectiveness. CGM did improve outcomes compared to patients who had never used a monitor. The control of HbA1c is largely influenced by compliance. The research objects included in this meta-analysis were biased. CGM was not popular at that time, and patients were more concerned about the cost of CGM. Our study incorporates recent high-quality randomized controlled trials that provide strong evidence for the results 22258980.

There are some limitations to our study. First, there was heterogeneity at the HbA1c level in the literature we included in the analysis. We have not been able to identify the source of heterogeneity. Second, the metrics we use to evaluate efficacy are inadequate, and more clinical indicators are needed to evaluate the efficacy of the two methods.

In conclusion, the results of this study suggested that continuous blood glucose monitoring is associated with lower blood glucose levels than the traditional blood glucose self-test method. Therefore, for patients with type 1 diabetes, CGM is a better method for monitoring blood glucose. It is suggested that type 1 diabetes patients, especially those with poor diabetes control, should use CGM instead of SMBG in blood glucose monitoring. This study promotes the management of patients with type 1 diabetes by evaluating the effectiveness of CGM and providing a reference for current and future related research.

## Figures and Tables

**Figure 1:** Document screening process and results.

**Figure 2:** HbA1c horizontal forest map. CGM: continuous glucose monitoring; SMBG: self-monitoring of blood glucose.

**Figure 3:** Horizontal funnel diagram of HbA1c. MD: mean difference.

**Figure 4:** Forest map of severe hypoglycemia events. CGM: continuous glucose monitoring; SMBG: self-monitoring of blood glucose.

**Figure 5:** Funnel diagram of severe hypoglycemia events. RR: risk ratio.

**Figure 6:** Forest chart of diabetes ketoacidosis. CGM: continuous glucose monitoring; SMBG: self-monitoring of blood glucose.

**Figure 7:** Funnel plot of diabetes ketoacidosis event. RR: risk ratio.

**Table 1:** Basic characteristics of included literature.

ID	Research type	Country	Blood glucose monitoring mode	Sample size	Insulin regimen	Age	Baseline HbA1c (mmol/mol)	Baseline HbA1c (%)	Diabetes mellitus time	Study time	Outcome indicators
Ajjan et al. 2016[10]	RCT	Britain	RT-CGM	28	MDI	39 ± 11.5	77.06 ± 14.21	9.2 ± 1.3	15.8 ± 11.9	100 days	HbA1c
			SMBG	13	MDI	43.7 ± 9.9	74.87 ± 14.21	9.0 ± 1.3	19.6 ± 12.4		
Beck et al. 2017[11]	RCT	U.S.	RT-CGM	105	MDI	46 ± 14	70.5 ± 7.65	8.6 ± 0.7	19.0 ± 14.8	24 weeks	HbA1c, SH, DKA
			SMBG	53	MDI	51 ± 11	70.5 ± 6.56	8.6 ± 0.6	21.7 ± 17.8		
Bolinder et al. 2016[12]	RCT	Europe	isCGM	120	MDI/CSII	42 ± 13.3	50.7 ± 5.7	6.79 ± 0.52	20.0 ± 10.4	24 weeks	HbA1c, SH, DKA
			SMBG	121	MDI/CSII	45 ± 17.8	50.6 ± 6.7	6.78 ± 0.64	21.3 ± 14.8		
Bosi et al. 2019[13]	RCT	Britain	RT-CGM	76	CSII	49.0 ± 12.2	60.7 ± 9.9	7.7 ± 0.9	28.5 ± 11.1	24 weeks	HbA1c, SH, DKA
			SMBG	77	CSII	47.4 ± 12.5	59.7 ± 9.9	7.6 ± 0.9	29.7 ± 13.3		
Boucher et al. 2020[14]	RCT	New Zealand	isCGM	33	MDI/CSII	16.5 ± 1.9	94.55 ± 18.58	10.8 ± 1.7	7.0 ± 3.5	24 weeks	HbA1c, SH, DKA
			SMBG	31	MDI/CSII	16.7 ± 2.2	98.92 ± 17.49	11.2 ± 1.6	8.0 ± 4.0		
Dicembrini et al. 2020[15]	Cross design test	Europe	RT-CGM	14	CSII	45.7 ± 8.2	60.66 ± 4.37	7.7 ± 0.4	17.3 ± 18.5	16 weeks	HbA1c, SH, DKA
			SMBG	14	MDI	44.7 ± 8.7	61.75 ± 5.47	7.8 ± 0.5	19.0 ± 19.3		
Heinemann et al. 2018[16]	RCT	Europe	RT-CGM	74	MDI	45.8 ± 12.0	59.57 ± 10.93	7.6 ± 1.0	20.9 ± 14.0	26 weeks	HbA1c
			SMBG	74	MDI	47.3 ± 11.7	57.38 ± 10.93	7.4 ± 1.0	21.6 ± 13.9		
Jensen et al. 2022[17]	RCT	Europe/North America	P-CGM	117	MDI/CSII	49 ± 12	58.2 ± 5.7	NR	28 ± 12	16 weeks	HbA1c, SH
			SMBG	355	MDI/CSII	42 ± 15	58.4 ± 5.9	NR	23 ± 12		
Laffel et al. 2020[18]	RCT	U.S	RT-CGM	74	MDI/CSII	17 ± 3	73.78 ± 10.93	8.9 ± 1.0	9.0 ± 5.0	26 weeks	HbA1c, SH, DKA
			SMBG	79	MDI/CSII	18 ± 3	73.78 ± 10.93	8.9 ± 1.0	10.0 ± 5.0		
Lind et al. 2017[19]	Cross design test	Europe	RT-CGM	82	MDI	46.7 ± 13	69.3 ± 9.84	8.49 ± 0.9	23.4 ± 11.9	26 weeks	HbA1c, SH, DKA
			SMBG	79	MDI	42.6 ± 12.2	68.86 ± 9.84	8.45 ± 0.9	21.0 ± 11.7		
Pratley et al. 2020[20]	RCT	U.S	RT-CGM	103	MDI/CSII	68.3 ± 5.2	59.57 ± 9.84	7.6 ± 0.9	37.3 ± 18.5	24 weeks	HbA1c, SH, DKA
			SMBG	100	MDI/CSII	67.3 ± 5.2	58.48 ± 8.74	7.5 ± 0.8	36.0 ± 16.3		
Thabit et al. 2020[21]	Cross design test	Britain	RT-CGM	16	MDI/CSII	21 ± 2.28	NR	NR	NR	8 weeks	HbA1c, SH, DKA
			SMBG	15	MDI/CSII	21.4 ± 2.57	NR	NR	NR		
Tumminia et al. 2015[22]	Cross design test	Europe	RT-CGM	10	MDI/CSII	NR	69.84 ± 4.37	8.54 ± 0.4	NR	24 weeks	HbA1c, SH, DKA
			SMBG	10	MDI/CSII	NR	NR	8.56 ± 0.5	NR		
van Beers et al. 2016[23]	Cross design test	Netherlands	RT-CGM	26	MDI/CSII	NR	NR	NR	NR	16 weeks	HbA1c, SH, DKA
			SMBG	26	MDI/CSII	NR	70.06 ± 5.47	NR	NR		
Zhang et al. 2021[24]	RCT	China	FGM	71	MDI/CSII	36.68 ± 19.71	NR	9.05 ± 1.43	4 ± 2.3	48 weeks	HbA1c
			SMBG	75	MDI/CSII	35.19 ± 18.91	NR	9.07 ± 1.18	5 ± 2.3		

Note: RT-CGM: real-time blood glucose monitoring; SMBG: self-blood glucose monitoring; isCGM: intermittent scanning CGM; P-CGM: individual continuous blood glucose monitoring; FGM: rapid blood glucose monitoring; SH: severe hypoglycemia; DKA: diabetes ketoacidosis; CSII: insulin pump; MDI: multiple subcutaneous injections per day; RCT: randomized control trials.

## Data Availability

The data used to support the findings of this study are available from the corresponding author upon request.
